# *Eafs* Control Erythroid Cell Fate by Regulating *c*-*myb* Expression through Wnt Signaling

This article has been retracted.

**DOI:** 10.1371/journal.pone.0064576

**Published:** 2013-05-22

**Authors:** Xufa Ma, Jing-Xia Liu

**Affiliations:** 1 College of Fisheries, Huazhong Agricultural University, Wuhan, P. R. China; 2 Institute of Hydrobiology, Chinese Academy of Sciences, Wuhan, P. R. China; New York Medical College, United States of America

## Abstract

ELL associated factor 1 and ELL associated factor 2 (EAF1/2 factors) are reported to play important roles in tumor suppression and embryogenesis. Our previous studies showed that *eaf* factors mediated effective convergence and extension (C&E) movements and modulated mesoderm and neural patterning by regulating both non-canonical and canonical Wnt signaling in the early embryonic process. In this study, through knockdown of both *eaf1* and *eaf2* in embryos, we found that differentiation of primary erythroid cells was blocked, but hematopoietic precursor cells maintained in *eaf*s morphants. Co-injection of *c-myb*-MO rescued the erythroid differentiation in *eaf*s morphants, as indicated by the restored expression of the erythroid-specific gene, *βe3 globin*. In addition, low dosage of *c-myb* effectively blocked the *βe3 globin* expression in embryos, and did not affect the expression of markers of hematopoietic progenitor cells and other mesoderm, which was similar to the phenotypes we observed in *eaf*s morphants. We also revealed that knockdown Wnt signaling by transiently inducing *dn-Tcf* in embryos at the bud stage down-regulated the increased *c-myb* to normal level and also restored *βe3 globin* expression in *eaf*s morphants. Our evidence points to a novel role for *eaf* factors in controlling erythroid cell fate by regulating *c-Myb* expression through canonic Wnt signaling.

## Introduction

Human hemoglobinopathies are a group of genetic disorders caused by abnormal expression of globin genes, that result in anemia in patients. The molecular mechanism underlying the globin genes induction is evolutionarily conserved among vertebrates, and the process appears to depend on the extensive sharing of lineage-restricted transcriptional factors [1]. *Gata1* is the erythroid factor, which is highly expressed in megakaryoytic/erythroid progenitors [2], [3], [4], [5]. It is essential for erythroid specification and differentiation [3], [5] and cooperates with *runx1* and *fli1*, which are involved in the divergence of megakaryoytic from the erythroid lineage [6], [7]. On the contrary, *Pu.1*, a myeloid factor, is lineage-restrictedly required for granulocyte/macrophage induction [2], [5]. *Lmo2*, *gata2* and *scl* are required earlier in the hematopoiesis process and restrict hemoto-vascular development of lateral mesoderm [8], [9]; in addition, they are also in a complex required for full erythroid cell maturation [10].

The *c*-*Myb* transcriptional factor is a key regulator of the hematopoietic stem and progenitor cells, one that is essential for the establishment of hematopoiesis as evidenced by the defects in the development of multiple blood lineages in the *Myb* null mice [11], [12], [13]. Conditional *c-Myb* knockout in adult hematopoietic stem cells leads to loss of self-renewal due to impaired proliferation and accelerated differentiation [14]. The *c-Myb* level must be down-regulated in order for hematopoietic cells terminal differentiation and maturation [15]. Constitutive expression of *c-Myb* blocks Friend murine erythroleukemia cell differentiation [16]. Expression of *c-Myb* was repressed by GATA-1 to allow further differentiation of erythrocyte at the onset of terminal differentiation in erythroblast [17], [18]. On the contrary, by using microRNAs to knockdown *c-Myb* expression in primary human erythroid progenitor cells, fetal and embryonic hemoglobin genes displayed elevated expression. This suggests that *c-Myb* plays an important role in silencing the fetal and embryonic hemoglobin genes [19]. In addition, those microRNAs elevate fetal hemoglobin expression via *c-Myb* in human trisomy13 [19].

During zebrafish embryogenesis, *eaf* factors have been revealed to mediate effective C&E movements through maintaining expression of non-canonical Wnt signaling ligands, Wnt5 and Wnt11 [20], and to modulate mesoderm and neural patterning by inhibiting canonical Wnt signaling [21]. In addition, *eaf* factors form a negative loop with another non-canonical Wnt signaling ligand, Wnt4, in embryos and mammalian cell lines [22]. In the embryos with morpholina-mediated *eaf1* and *eaf2* knockdown, we observed the high percentage of erythroid differentiation defects, but we still know little about the underlying mechanisms.

In this study, by screening potential repressors of erythroid differentiation in *eaf*s morphants using morpholino-mediated knockdown, we selectively and respectively co-injected morpholinos of genes that had been reported to inhibit erythroid differentiation and also displayed increased expression in *eaf*s morphants. By co-injecting with *c-myb*-MO [23], we found that knockdown *c-myb* in *eaf*s morphants could effectively rescue the erythroid differentiation defects, indicated by restored *βe3 globin* expression. Consistently, an over-expressed *c-myb* in embryos could nearly phenocopy the erythroid differentiation defects shown in *eaf*s morphants. In addition, in *eaf*s morphants, by transiently inducing *dn*-*Tcf*, a dominant negative form of Wnt signaling, we found that knockdown of canonical Wnt signaling can not only restore the increased expression of *c-myb* to normal levels, but also restore the reduced *βe3 globin* expression. In our study, we reveal a novel genetic cascade in the process of erythroid differentiation, in which Wnt signaling up-regulates expression of hematopoietic progenitor-restricted transcriptional factors, including *c-myb*, and the increased *c-myb* mediates the suppression of erythroid differentiation.

## Materials and Methods

### Fish Stocks

As previously discussed, wild-type zebrafish (*Danio rerio*) (AB) maintenance, breeding, and staging were performed [20] and the hs:dnTCF-GFP transgenic line was performed as reported previously [24], [25].

### Heat-shock Modulation

Embryonic heat-shock experiments were conducted at 38°C for 20 minutes. Genotype was determined by the presence of GFP fluorescence at 3 hours post heat shock, then the non-fluorescent (wild-type) siblings were sorted and used as controls [24], [25].

### Morpholino and mRNA Synthesis

The translation blocking morpholinos (ATG targeted) *eaf1*-MO1 and *eaf2*-MO1, and splicing-blocking morpholinos, *eaf1*-MO3 and *eaf2*-MO3, have been described previously [20], [21], as the *c-myb* antisense morpholino have been described previously [23]. All morpholinos were purchased from Gene Tools, LLC (Philomath, Oregon, USA) and their sequences are listed in Table S1.

For mRNA preparation, capped mRNA of *c-myb* was synthesized using the Ampticap SP6 High Yield message maker kit (Epicenter Biotechnologies). The synthesized mRNAs were diluted into different concentrations and injected into one-cell stage embryos, and the plasmid for *c-myb* mRNA was described previously [26].

### Whole Mount *in situ* Hybridization and O-Dianisidine Staining

Probes for *gata2*, *fli1*, *scl*, *lmo2*, *runx1*, *gata1*, *pu.1*, *c-myb* and *flk1* were reported previously [3], [26], [27]. Probes for *pax2a* and *myoD* were kindly provided by Dr. Schier (Harvard University, Molecular and Cellular Biology), probe for *cdh5* was kindly provided by Dr. Wang (Institute of Hydrobiology, Chinese Academy of Science), and probe for *ntl* was reported previously [20]. The procedures for *in situ* hybridization and o-dianisidine staining were performed as described previously [20], [28].

### Western Blot

Western blot was performed as described previously [29]. The embryos at the 24 hpf were washed with ice-cold PBS buffer and then lysed in RIPA (radioimmune precipitation) buffer containing 50 mM Tris, pH 7.4, 1% NP-40, 0.25% Na-deoxycholate, 1 mM EDTA, pH 8.0, 150 mM NaCl, 1 mM NaF, 1 mM PMSF (phenylmethylsulphonyl fluoride), 1 mM Na_3_VO_4_ (sodium orthovanadate) and 1∶100 dilution of protease inhibitor cocktail (Sigma). After homogenizing, lysates were centrifuged for 15 minutes at 12,000 g at 4°C, and the supernatants were boiled with 1× SDS sample buffer, separated on SDS-PAGE and transferred to PVDF membrane (Millipore). The Western blot analysis was performed as described previously using the indicated anti-*βe3 globin* antibody (Z-Fish™ (Zebrafish)) and anti-β-actin antibody (Abcam).

## Results

### *Eafs* are Required for Erythroid Differentiation

In our previous studies, we observed C&E movement defects and forebrain defects in *eaf1* and *eaf2* morphants, revealing that both *eaf1* and *eaf2* mediate C&E movements by non-canonical Wnt signaling and modulate mesoderm and neural patterning by inhibiting canonical Wnt signaling [20], [21]. In the late stage, in *eaf*s morphants at 2 dhf, we observed significant defects including heart edema, reduced circular blood cells, and a lack of blood flow or clumps of blood cells located in front of the beating heart in embryos knockdown both of *eaf1* and *eaf2* (data not shown), suggesting that the *eaf*s morphants displayed hematopoietic defects, as observed in *mll* morphants [30]. Here, in order to further test the molecular characters underlying the phenotypes, we applied blood markers to detect the hematopoietic defects in *eafs* morphants.

Knockdown of both *eaf1* and *eaf2* in embryos by injection of either translation-blocking ATG-MO (indicated by *eaf*s-MO1, and shown in Figure 1) or “splicing-blocking” morpholinos (data not shown) caused a striking hematopoietic phenotype. Morpholinos reduced functional *eaf*s message, yielded obviously erythroid defects (Figure 1). Hemoglobin, indicated by o-dianisidine staining, reduced significantly in *eaf*s morphants (Figure 1, A2, A3 and A4) compared to its control group (Figure 1, A1, A3 and A4), and nearly 100% of morphants displayed dramatically reduced differentiated mature erythrocytes (Figure 1, A3 and A4). By whole mount *in situ* hybridization (WISH), transcripts of *βe3 globin*, which marked mature erythroid, displayed obviously reduced expression in over half of the detected *eaf*s morphants (59 of 95 morphants, Figure 1, B2); its protein level also reduced significantly in *eaf*s morphants compared to its expression in control embryos (Figure 1, C).

**Figure 1:** *Eaf*s are required for specification of erythroid cells. (A) Erythroid defects in *eaf*s morphants were detected by o-dianisidine staining for hemoglobin. (B) *Eafs* morphants displayed erythroid defects, indicated by reduced mRNA of *βe3 globin*. (C) *Eaf*s morphants displayed reduced protein of *βe3 globin*.

### Erythroid Defects in *Eaf*s Morphants are Specific

To determine the specificity of *eaf*s-MO induced erythroid defects, we examined the integrity of non-hematopoietic tissues and other markers which labeling vasculature and hematopoietic progenitors (Figure 2). *Eaf*s morphants displayed obviously anterior neuroectoderm truncation at 24 hpf (Figure 2, A2 and A4, indicated by black arrowhead). These observations were consistent with our previous report that *eaf*s were required for forebrain formation [21]. But the posterior mesoderm, including muscle and notochord, at 24 hpf, were intact but displayed subtle patterning defects in *eaf*s morphants. *MyoD* displayed more compact expression and striped muscles was irregular (Figure 2, A2), it might be a phenotype of C&E movement defects as we observed previously [20]. Notochord (*ntl*: Figure 2, A3 and A4) was also normal in a representative morphant which displayed severe anterior truncation (Figure 2, A4, anterior truncation is indicated by black arrowhead). Functional vasculature and primitive hematopoietic progenitors were normal and maintained in *eaf*s morphants. By WISH, *eaf*s-MO injected embryos had a few increased progenitors (*c-myb*: A5, A6; *scl*: A7, A8, indicated by black arrow), and had increased vasculature (*chd5*; A9, A10; *flk1*; A11, A12).

**Figure 2:** Erythroid defects in *eaf*s morphants are specific. (A) At 24 hpf to 26 hpf, the expression detection of control or *eaf*s-MO injected embryos (8 ng per embryo) processed by WISH for tissue specific genes: somites (A1, A2), notochord (A3, A4), vasculature (*cdh5*: A9, A10; *flk1*: A11, A12), and primitive progenitors (*c-myb*: A5, A6; *scl*: A7, A8, indicated by black arrow). (B) At the 8 somites stage, primitive hematoposis in *eaf*s morphants, indicated by primitive progenitor genes (*scl*: B1, B2; *lmo2*: B3, B4). (C) At the 10 somites stage, progenitors for blood (*gata2*: C1, C2; *lmo2*: C3, C4; *runx1*: C7, C8; *c-myb*: C15, C16), progenitors for vasculature (*fli*: C11, C12), progenitors for both blood and vasculature (*scl*: C5, C6), more mature erythroid progenitors (*gata1*: C9, C1**0**), and more mature myeloid progenitors (*Pu.1*: C13, C14). A1–A12, C13–C16, lateral view, anterior to the left. B1–B4, C1–C12, dorsal view, anterior to the up.

In order to test whether the initiation and progress of primitive hematopoiesis were normal in *eaf*s morphants, we detected blood progenitor-restricted transcriptional factors during early somitogenesis. At the 8 somites stage, blood progenitors indicated by *scl* (Figure 2, B1 and B2), which is required earlier in the hematopoiesis and is important for both blood and vessel development, showed normal in *eaf*s morphants. Similarly, *lmo2*, another important transcriptional factor required earlier in the hematopoiesis process and restricting hemoto-vascular development of lateral mesoderm, also displayed normal in *eaf*s morphants (Figure 2, B3 and B4). When the morphants developed to the 10 somites stage (Figure 2, C), however, there was a little overexpression in *scl* (Figure 2, C5 and C6), and *lmo2* (Figure 2, C3 and C4), compared to their respective control; *Gata2* (Figure 2, C1 and C2), *runx1* (Figure 2, C7 and C8), and *pu.1* (Figure 2, C13 and C14) displayed increased expression in *eaf*s morphants from the 10 somites stage; A slight overexpression was also observed in case of *fli* (Figure 2, C3 and C4), *gata1* (Figure 2, C9 and C10), and *c-myb* (Figure 2, C15 and C16).

### Knockdown *C-myb* in *Eaf*s Morphants Restored *βe3 globin* Expression

The above observations indicated that blood precursor-restricted transcriptional factors, including *gata2*, *fli*, *scl*, *runx1*, *gata1*, *lmo2*, *pu.1*, and *c-myb* increased in *eaf*s morphants from the 10 somites stage (Figure 2), but *βe3 globin* reduced dramatically (Figure 1). *Gata1* is essential for erythroid cell fate determination [3], [5], and *gata2*, *scl*, and *lmo2* are factors in the transcriptional complex for erythroid maturation [8], [9], [10]. However, *pu.1*, *runx1*, *fli*, and *c-myb* are negative factors that antagonize erythroid differentiation and maturation [6], [7]. Thus, we analyzed whether the reduced *βe3 globin* expression might result from the up-regulation of *pu.1*, *runx1*, *fli*, or *c-myb* in *eaf*s morphants. In order to investigate this hypothesis further, we performed morphorlino-mediated knockdown of those transcriptional factors in *eaf*s morphants respectively. We found that knockdown of *c-myb* could restore *βe3 globin* expression in *eaf*s morphants to some extent (Figure 3, A3), far fewer embryos (22 of 86 specimen) displayed reduced *βe3 globin* expression after co-injected with *c-myb*-MO (Figure 3, A3) compared to *eaf*s signal morphants (51 of 95 specimen) (Figure 3, A2). In addition, *βe3 globin* expression also increased in rescued embryos compared to its level in *eaf*s morphants (Figure 2, A3).

**Figure 3:** *Eaf*s act upstream of *c-myb* in primitive hamatopoiesis. (A) In situ hybridization of *βe3 globin* showing rescue of erythroid differentiation defects in *eaf*s morphants by knockdown of *c-myb*, the numbers of embryos displayed reduced *βe3 globin* in total detected embryos was shown in (A2, A3). (B) *βe3 globin* expression in *eaf*s morphants (B2) and in,*c-myb* morphants (4 ng per embryo) (B3) and in morphants injected with combined *eaf*s-MO and *c-myb*-MO (8 ng *eaf*s-MO per embryo and 2 ng *c-myb*-MO) (B4). (C) Morphology of representative embryos injected with *c-myb*-MO (C2), and mesoderm pattern indicated by expression of *pax2a* and *myoD* in *c-myb* morphants at the bud stage (C4). (D) *C-myb* function downstream of *eaf*s in primitive hematopoiesis. Early hematopoietic progenitors, *lmo2*, displayed obviously reduced expression from the 6 somites stage both in *c-myb* morphants (4 ng per embryo) (D2) and in morphants injected with combined *c-myb*-MO and *eaf*s-MO (8 ng *eafs*-MO/per embryo and 2 ng *c-myb*-MO) (D3). *Gata1* and *scl* also displayed obviously reduced expression in embryos injected with combined *eaf*s-MO and *c-myb*-MO (D6, D9) as in embryos injected with *c-myb*-MO single (D5, D8) at the 10 somites stage. A1–A3, D1–D9, dorsal view, anterior to the up; C3, C4, dorsal view, anterior to the left. B1–B4, C1, C2, lateral view, anterior to the left.

Contrary to *eaf*s morphants (Figure 3, B2), *c-myb* morphants displayed little elevation of expression of *βe3 globin* (Figure 3, B3); the morphants injected with both *eaf*s-MO and *c-myb*-MO displayed in-between expressions of *βe3 globin* (Figure 3, B4). We also analyzed the morphogenesis of *c-myb* morphants and defects of non-blood mesoderm in *c-myb* morphants. As shown in Figure 3C, the *c-myb* morphants displayed similar phenotypes to those reported previously such as small eyes and small brain (Figure 3, C2) [23], but no obvious defects displayed in the posterior body. In *c-myb* morphants, the induction of non-blood mesoderm, indicated by *pax2a* and *myoD*, also displayed normal expression at the bud stage, although there appear to be subtle patterning defects such as short *myoD* domain in *c-myb* morphants (Figure 3, C4).

### *C-myb* was Required for Maintaining of Hematopoietic Precursors

Although we found that knockdown *c-myb* in *eaf*s morphants could rescue *βe3 globin* expression effectively, we still knew little about the genetic cascade between *c-myb* and *eaf* factors in this process. In order to further understand the genetic pathway between *c-myb* and *eaf* factors in hematopoiesis, we detected more blood markers in *c-myb* morphants and in morphants co-injected with *c-myb*-MO and *eaf*s-MO together.

In PLM (posterior lateral mesoderm), the initiation of *c-myb* was detected around the 4 somites stage [31], [32], so we detected the expression of blood markers in *c-myb* morphants from the 6 somites stage. As shown in Figure 3D, the expression of *lmo2* reduced significantly in *c-myb* morphants from the 6 somites stage (27 of 27 specimen, Figure 3, D2). In embryos co-injected with both *c-myb*-MO and *eaf*s-MO, *lmo2* displayed obviously reduced expression (10 of 13 specimen, Figure 3 D3). In addition, *gata1* (14 of 15 specimen, Figure 3, D5) and *scl* (19 of 21 specimen, Figure 3, D8) also displayed dramatically reduced expression in *c-myb* morphants. Similarly, in embryos injected with both *c-myb*-MO and *eaf*s-MO, *gata1* (8 of 10 specimen, Figure 3, D6) and *scl* (13 of 15 specimen, Figure 3, D9) also displayed reduced expression, as we observed in *c-myb* morphants. All the observations suggested that *c-myb* might be required to maintain the hematopoietic progenitor cells and could also act downstream of *eaf*s in specification blood cells or regulating expression of blood transcriptional factors.

### *C-myb* Suppressed *βe3 globin* Expression, but Had no Influence on Hematopoietic Precursors

With all the above observations taken together, we assumed that *c-myb* might be required for hematopoietic precursor cells, but would block erythroid differentiation in zebrafish, thus functioning similarly with its mammalian orthologs [14], [17], [19]. To further detect its roles in hematopoiesis *in vivo*, we over-expressed *c-myb* in embryos by mRNA injection. We injected the embryos with different dosages of *c-myb* mRNA, from 50 pg per embryo to 200 pg per embryo, and the embryos did not display defects of morphology (data not shown). We analyzed the development of hematopoietic cells in embryos injected with different dosages of *c-myb* mRNA respectively. Most embryos injected with *c-myb* mRNA displayed obviously reduced expression of *βe3 globin*, either the dosage was 50 pg per embryo (Figure 4, A2) or was 200 pg per embryo (Figure 4, A4), however, *gata1*, displayed normal expression in all the detected embryos injected with different dosages of *c-myb* mRNA (Figure 4, A6 and A8). The observations here suggested that, *c-myb* could effectively suppress *βe3 globin* expression *in vivo* even at a very low dosage (50 pg per embryo). In order to further detect the roles of *c-myb* in hematopoiesis in zebrafish embryos, we detected more molecular markers labeling non-hematopoietic tissues or hematopoietic cells, with all embryos injected with the same dosage of *c-myb* mRNA (50 pg per embryo). At this low dosage (50 pg per embryo), *c-myb* could effectively suppress *βe3 globin* expression *in vivo* (37 of 70 specimen, Figure 4, B2), and the corresponding injected *c-myb* mRNA displayed ubiquitously distribution (Figure 4, B4). We wondered whether reduced *βe3 globin* expression resulted from mesoderm pattern defects, then we detected the expression of other molecular markers, including markers labeling hematopoietic precursors and axis mesoderm, in embryos with ectopic *c-myb* expression (50 pg per embryo). At the 10 somites stage, the erythroid precursor marker, *gata1*, displayed similar expression levels in embryos with ectopic expression of *c-myb* (Figure 4, C2) as in control embryos (Figure 4, C1). Similarly, *scl*, another erythroid precursor marker, also displayed normal expression in embryos injected with *c-myb* mRNA (Figure 4, C3 and C4). In addition, non-blood mesoderm markers, *pax2a* and *myoD*, showed normal expression in embryos with ectopic *c-myb* expression (Figure 4, C6) when compared to control embryos (Figure 4, C5). All the data suggested that *c-myb* specifically inhibited *βe3 globin* expression, but had no influence on expression of axis mesoderm and hematopoietic precursor cells in embryos.

**Figure 4:** *C-myb* suppressed specification of mature erythroid cells, and the phenotype of *c-myb* gain of function is specific. (A) Different dosage of *c-myb* on specification of mature erythroid cells (*βe3 globin*: A2, 50 pg per embryo; A4, 200 pg per embryo) and on erythroid progenitors (*gata1*: A6, A8). (B) *In situ* hybridization of *βe3 globin* showed that erythroid differentiation was blocked in embryos with ectopic *c-myb* expression (50 pg per embryo) (B2), the number of embryos displayed reduced *βe3 globin* was shown in (B2), and the *in situ* hybridization of *c-myb* shown its ectopic expression in corresponding embryos (B4). (B) Hematopoietic progenitor cells including *gata1* (C1, C2) and *scl* (C3, C4), and other mesoderm cells including *pax2a* and *myoD* (C5, C6) specified and maintained normally in embryos with ectopic *c-myb* expression. A1–A8, B1, B2, C1–C4, dorsal view, anterior to the up; B3, B4, C5, C6, lateral view, anterior to the left.

### *Eaf* Regulate Erythroid Cell Differentiation by Modulating *C-myb* Expression through Wnt Signaling

The above observations suggested that the increased expression of *c-myb* might mediate the suppression of erythroid differentiation in *eaf*s morphants. High Wnt signaling was revealed in *eaf*s morphants [21], and Wnt signaling was reported as being required for stem cell renewal and for inhibiting terminal multi-linage cells differentiation [33], [34], [35]. In addition, down-regulating Wnt activities resulted in significantly reduced expression of *gata1* in intermediate cell mass (ICM) [36], and *c-myb*, in aorta-gonad- mesonephros (AGM) [25], in treated embryos.

In this study, by applying hs:dnTCF-GFP transgenic embryos [24], [25], [36], which is a stable line that express a dominant negative of TCF/LEF, we down-regulated Wnt activities by transiently induceing *dn-Tcf* expression in embryos, and detected some hematopoietic cell markers including *gata1*, *c-myb* and erythroid specific markers. The scheme of knockdown Wnt signaling in embryos using hs:dnTCF-GFP fish was shown in Figure 5A. We heat-shocked the embryos at the bud stage, there was no obvious morphology defects observed in the GFP positive embryos at the 16 somites stage or later (data not shown), which differs from the previous report that the embryos showed malformation after heat-shocking at 75% epiboly stage [36]. We detected the expression of hematopoietic precursors and erythroid markers in *dn-Tcf* transgene induced embryos. Compared to their control offsprings (Figure 5, B1 and B3), embryos with expression of transiently induced *dn-Tcf*, both *c-myb* (Figure 5, B2) and *gata1* (Figure 5, B4) displayed obviously reduced expression, the observations here were consistent with previous reports [25], [36].

**Figure 5:** Knockdown Wnt signaling in hs:dnTCF-GFP embryos by heat shock at the bud stage resulted in reduced progenitor cells and accelerated differentiation of erythroid cells. (A) Scheme of using hs:dnTCF-GFP fish to knockdown Wnt signaling in embryos. (B) Reduced progenitor blood cells, labeled by *c-myb* (B1, B2) and *gata1* (B3, B4), but accelerated erythroid cells differentiation, labeled by *βe3 globin* (B5, B6, B9, B10) and *band3* (B7, B8) displayed in hs:dnTCF-GFP positive embryos, and black arrow indicate the increased expression of *βe3 globin* expression in hs:dnTCF-GFP positive embryos (B10) compared to its control siblings (B9). Other mesoderm, labeled by *pax2a* and *myoD* (B9, B10, B11, B12), was normal in hs:dnTCF-GFP positive embryos. B1, B2, B7–B12, lateral view, anterior to the left; B3–B6 dorsal view, anterior to the up.

The differentiated erythroid markers, *βe3 globin* (Figure 5, B6 and B10) and *band3* (Figure 5, B8),however, showed small increase in the embryos with induced *dn-Tcf* expression. We could not detect the expression change of non-blood axis mesoderm, such as *pax2a* and *myoD*, in the embryos with transiently induced *dn-Tcf* expression (Figure 5, B11 and B12), consistent with the observations that no obvious morphology defects displayed in the heat-shocked GFP positive embryos (data not shown).

We then contemplated whether down-regulating Wnt signaling in *eaf*s morphants could rescue the erythroid defects and down-regulate the expression of precursor markers. Figure 6A shows the scheme of using hs:dnTCF-GFP fish to do rescue experiments. As expected, transiently inducing expression of *dn*-*Tcf* in *eaf*s morphants could restore the expression of *βe3 globin* significantly (Figure 6, B and C). In a total of 27 *eaf*s morphants, 48.2% of morphants displayed strongly reduced *βe3 globin* expression, 22.2% of morphants displayed mildly reduced *βe3 globin* expression, and 29.6% of morphants shown normal (Figure 6, C); but after heat-shocking to induce *dn-Tcf* expression in *eaf*s morphants, we found that in a total of 29 detected embryos, only 6.9% of morphants showed strongly reduced expression of *βe3 globin*. Another 34.5% of morphants even shown increased expression of *βe3 globin* (Figure 6, B and.C), suggesting that *dn*-*Tcf* might act downstream of *eaf*s and be very effective to rescue differentiation defects of erythroid cells in *eaf*s morphants. In addition, the increased expression of *c-myb* was also restored to a normal level by transiently inducing *dn-Tcf* expression in *eaf*s morphants (Figure 6, B and C).

**Figure 6:** Knockdown Wnt signaling in *eaf*s morphants by transiently inducing *dn-Tcf* expression rescued defects of *c-myb* expression and erythroid cells specification. (A) Scheme of rescuing experiments in *eaf*s morphants by using hs:dnTCF-GFP embryos. (B) Increased *c-myb* expression and reduced *βe3 globin* expression were restored in *eafs* morphants by transiently inducing *dn-Tcf* in embryos at the bud stage. B1–B8, dorsal view, anterior to the up.

## Discussion

### Erythroid Differentiation is Blocked in *Eaf*s Morphants, and the Phenotype is Specific

*Eaf* factors play important roles in tumor suppression and embryogenesis. In zebrafish, by morpholino-mediated knockdown, we revealed that *eaf* patterned the embryonic axis by regulating both non-canonical and canonical Wnt signaling at early developmental stages [20], [21]. At later stages, we observed significant defects including reduced circular blood cells and a lack of blood flow in *eaf*s morphants. By further detecting the molecular markers of hematopoietic cells in *eaf*s morphants, obvious defects of erythroid differentiation were revealed, indicated by reduced mRNA and protein level of *βe3 globin* and significant reduced o-dianisidine staining hemoglobin in *eaf*s morphants (Figure 1). Normal vasculature (Figure 2, A9–A12), the integrity of posterior non-hematopoietic tissues indicated by *myoD* and *ntl* (Figure 2, A1–A4), and increased expression of precursors of blood and vessel, indicated by increased expression of *gata1*, *scl*, *lmo2*, *gata2*, *pu.1*, *runx1*, *fli1*, and *c-myb* in *eaf*s morphants from the 10 somites stage (Figure 2, A5–A8 and C), both suggested that defects of erythroid specification in *eaf*s morphants were highly specific and not due to the expense of nearby tissues. Morphants at 24 hpf displayed severe anterior truncation (Figure 2, A2 and A4, indicated by black arrowhead), the observations here were consistent with our previous reports that *eaf*s are required for forebrain formation in embryos [20], [21], [22]. In *eaf*s morphants, the specification and formation of the erythroid progenitors were normal, but erythroid differentiation was blocked, suggested that the cells in the primary hematopoietic process might keep and accumulate on the precursor stage. The following observations help to support this point.

Firstly, in our study, all precursor markers, including *gata1*, *scl*, *lmo2*, *gata2*, *c-myb* and other genes, displayed increased expression from the 10 somites stage (Figure 2, A and C), but their expressions were still normal, even when detected by the 8 somites stage (Figure 2, B), and it was impossible that some factors could generally up-regulate all the precursor markers in such a short time. Second, it is reported that the initiation of erythroid began around the 8–10 somites stage in zebrafish embryos [37] (personal communication with Jared J. Ganis). In our study, the increased expression of precursor markers began shortly after the initiation of erythroid differentiation (Figure 2, B and C), this might only happen after the blocking of erythroid differentiation. If we could count the whole number of blood cells and the ratio of precursor cells and differentiated erythroid cells in both control embryos and in *eaf*s morphants, we might perceive more clear mechanism clues underlying the phenotypes in *eaf*s morphants. Of course, we still could not remove the possibility that the increased expression of precursor markers might come from the accelerated proliferation of progenitor cells or from their increased expression in a single cell.

In *eaf2* knockout mice, Xiao et al also found hematopoiesis defects [38], [39]. Very small number of *eaf2* knockout mice developed extramedullary hematopoiesis, they suggested that *eaf2* inactivation may disrupt the normal hematopoiesis in bone marrow, causing a compensatory response from spleen and liver in the *eaf2* knockout mice [38], [39]. In addition, *eaf2* deletion enhanced B-cell lymphoma development in *eaf2* knockout mice [39], and *eaf1* and *eaf2* have been implicated in human hematopoietic cancers [40], [41]. Our data here showed more a detail character of the hematopoiesis defects cause by *eaf1* and *eaf2* knockdown *in vivo*, and the data here also suggested that the roles of *eaf* factors in regulating hematopoiesis might be conserved from zebrafish to mice.

### *C-myb* was Downstream of *Eaf*s in Hematopoietic Developmental Process

We observed increased expression of precursor markers but dramatically suppressed erythroid differentiation in *eaf*s morphants (Figure 1, Figure 2). Through a morphorlino-mediated knockdown of *c-myb* in *eaf*s morphants, we found that knockdown *c-myb* could significantly restore *βe3 globin* expression in *eaf*s morphants (Figure 3, A and B).

*C-myb* morphants displayed a morphogenesis phenotype as reported previously [23], characterized by a small brain but normal body axis formation (Figure 3, C2). Consistent with its normal formation of posterior body axis by morphology, we also observed normal pattern of mesoderm markers in *c-myb* morphants, indicated by *pax2a* and *myoD* expression (Figure 3, C4). But the primary hematopoietic wave failed in *c-myb* morphants, indicated by reduced expression of progenitor markers and accelerated erythroid differentiation before 24 hpf (Figure 3, B and D).

On the contrary, embryos with ectopic expression of *c-myb* displayed reduced expression of erythroid markers but normal expression of hematopoietic precursors in fish (Figure 4). It is reported that *c-Myb* is required for the development of hematopoietic precursors [12], [13], and conditional *c-Myb* knockout in adult hematopoietic stem cells leads to impaired proliferation and accelerated differentiation in mouse[14]. In addition, *c-Myb* suppresses erythroid differentiation [16] and plays an important role in silencing the fetal and embryonic hemoglobin genes [19]. Our data here supported that *c-myb* is required for maintaining hematopoietic precursor markers, but blocks erythroid differentiation, and suggests that the roles of *c-myb* in hematopoiesis were conserved from zebrafish to mammalian.

*C-myb* is a transcriptional factor which is important in hematopoiesis; it can bind with a vast number of different proteins in specifying different lineage of blood cells. The conditional *c-myb* knockout mice displayed hematopoietic defects in bone marrow [14], totally opposite to hematopoietic defects in a *c-myb* M303 mutant [42]. Similarly with the observations in mice, in this study, the hematopoietic defects occurred in *c-myb* morphants, which are different from what Thompson et al observed in *c-myb* b316 mutants; they found that *gata2*, *lmo2*, and *gata1* displayed normal expression in the mutants around 18 hpf [26]. We speculate, *c-myb* b316 mutants, similar to mice *c-Myb* M303 mutant, maybe only lost binding ability with some specific protein or lost some specific roles important for embryogenesis development, but its ability in regulating primary hematopoiesis still exists. The limitation of this mutant model can not truly or really tell us about the hematopoietic specification as the *c-myb* gene is disrupted by morpholino mediating knockdown in embryos. *C-Myb* specifically inhibited erythroid specification was convinced in this study (Figure 4), although we still know little about the underlying mechanisms. Countless literatures report that *c*-*Myb* is a myeloid lineage regulator, cooperates with C/EBPa, to activate transcription of myeloid genes [43], [44]. Recently, hematopoietic genes, especially myeloid other than erythroid genes, have been identified as direct targets of *c-Myb* by ChIP-Seq (chromatin immunoprecipitation followed by massively parallel sequencing) [45], [46]. Myeloerythroid lineage cells initiate expression of both myeloid and erythroid lineage regulator [2], and myeloid lineage regulator C/EBPa could compete with erythroid lineage regulator *gata1*, to shift binding of SMAD1 to sites of nonerythroid [47]. Since our observations showed that *c-myb* inhibited erythriod specification (Figure 3 and Figure 4), taken the above mentioned reports together, we suppose that, *c-myb* might act as a nonerythroid lineage regulator, compete with erythroid lineage regulator *gata1* or others, to bind with general master regulators, such as SMAD1, function indirectly in erythroid specification, However, we need more evidences to prove this speculation.

All the hematopoietic markers in *c-myb* morphants displayed the opposite expression pattern to their expression in *eaf*s single morphants (Figure 3, B and D). In morphants injected with *c-myb*-MO and *eaf*s-MO together, the hematopoietic precursors also reduced dramatically (Figure 3, D), similar to what we observed in *c-myb* morphants (Figure 3, D) but opposite to their expression in *eaf*s morphants (Figure 2, A and C). Combining the similarity of *βe3 globin* expression in *c-myb* morphants and in morphants knockdown with both *eaf*s-MO and *c-myb*-MO, but opposite to its expression in *eaf*s morphants together, we speculated that *c-myb* might act downstream of *eaf* factors in hematopoietic cells specification and differentiation.

### *Eaf* Control Erythroid Cell Fate by Regulating *C-myb* Expression through Wnt Signaling

*Eaf* factors have been revealed to modulate mesoderm and neural patterning by inhibiting canonical Wnt signaling, and high activity of canonical Wnt/β-catenin is revealed in *eaf*s morphants [21]. Wnt signaling was reported to be required for renewal of stem cells and progenitor cells and for inhibiting terminal multi-linage cells differentiation [33], [34], [35]. In addition, the expression of a hematopoietic precursor marker, *gata1*, reduced significantly in ICM in embryos with down-regulating Wnt activities [36].

In this study, we down-regulated Wnt activities in embryos by transiently induceing expression of *dn-Tcf* transgene, and revealed that including the reported gene *gata1* (Figure 5, B3 and B4) [36], other precursor markers, specially *c-myb* (Figure 5, B1 and B2) [25] and *pu.1* (data not shown), all displayed reduced expression. Our data was not only consistent with the previous study [25], [36], but also suggested that down-regulating Wnt activities in embryos could result in general down-regulating expression of most precursor markers. But how Wnt signaling acts on those cells in primitive hematopoiesis? Is this specific or direct? Since Goessling et al found that Wnt acts directly in AGM to promote hematopoietic stem cells proliferation [25], we need to evaluate how Wnt signaling act in blood forming regions in primitive hematopoiesis by applying one or more Wnt reporter lines in future days.

However, we could not detect any morphology defects under macroscopic detection (data not shown) or by staining of axis mesoderm markers (Figure 4, B11 and B12) in the treated embryos with transiently induced *dn-Tcf* expression. The reason for this might be that we treated embryos at the bud stage (Figure 4, A), and it is well-known that Wnt signaling has no influence on the axis pattern after 90% epiboly.

By transiently inducing *dn-Tcf* transgene expression, we rescued *βe3 globin* expression in *eaf*s morphants, and the increased *c-myb* expression was restored to normal level (Figure 6, B and C). Some morphants even showed increased expression of *βe3 globin* after heat-shocking (Figure 6, C), suggesting that *dn-Tcf* might act downstream of *eaf*s and be more efficient than *eaf*s in the determination and specification of erythroid cells.

As such, we elicit a model of hematopoietic process in *eaf*s morphants in which knockdown *eaf*s in embryos resulted in constitutive Wnt activities in the initiation and progress of hematopoietic cells specification and differentiation. The high Wnt activities induced increased expression hematopoietic precursor-restricted transcriptional factors, including *c-myb*, then the increased *c-myb* suppressed erythroid differentiation. Our data here also provided a novel mechanism that *c-myb* might mediate Wnt signaling in erythroid differentiation.

## Supporting Information

Table S1 **Morpholinos used in this study.**
(DOC)
